The article "Research Progress of B-Cell Lymphoma/Leukemia-2 Inhibitor Combined with Azacytidine in the Targeted Therapy of Acute Myeloid Leukemia" was retracted in 2023. Reasons: signs of a paper mill; suspected computer-generated content; unreliable results or conclusions; concerns about the data.

# Research Progress of B-Cell Lymphoma/Leukemia-2 Inhibitor Combined with Azacytidine in the Targeted Therapy of Acute Myeloid Leukemia

**DOI:** 10.1155/2022/3992224

**Published:** 2022-10-08

**Authors:** Yanyu Wang, Dan Huang, Lejia Liu, Aixin Wang, Yuan Gao, Huan Lin

**Affiliations:** Department of Oncology and Hematology, People's Hospital of Leshan, Leshan 614000, Sichuan Province, China

## Abstract

**Objective:**

To investigate the efficacy and safety of azacytidine and B-cell lymphoma/leukemia-2 inhibitors in the treatment of patients with acute myeloid leukemia (AML) and myelodysplastic syndrome (MDS).

**Methods:**

The clinical data of 31 patients with AML/MDS who were clearly diagnosed with AML/MDS were analyzed from 2018.10 to 2021.02, and the total amount of azacyclonol and B-cell lymphoma/leukemia-2 inhibitor was used for single or combined chemotherapy, with a total amount of 75 mg/m^2^^∗^7 d, divided into 7-10 days of continuous subcutaneous injection, every 28-30 days for a course of treatment. Overall response rate (ORR), median survival, poor response, and genetic mutations were observed.

**Results:**

A total of 104 courses of treatment were completed in 31 patients, the median course was 3 (1–12), and 6 patients who did not complete 2 courses of treatment were not counted in the statistics. After 2 courses, ORR was 72.0%, CRES was 2 (8.0%), mCR was 16 (64.0%), disease stable was 5 (20.0%), treatment failures were 2 (8.0%), mortality was 40.0%, and median survival time was >5 months. Single-agent and combined ORR was 64.3% and 81.8%, respectively, with median survival of 7.25 and 9 months; ORR for MDS and AML was 66.7% and 76.9%, respectively, median survival of 8 and 11 months was 66.7% and 80.0% of ORRs at 260 and V60 years, respectively, and median survival of 7 and 11.5 months; MDS-EB-1. The ORR of MDS-EB-2 was 75.0% and 62.5%, respectively, with median survival times of 11.5 and 6.5 months. During 2 courses and 4 courses, the rate of transfusion dependence was 64.0% and 55.5%, respectively. Fifteen cases were detected by second-generation sequencing, and the results were 14 cases of combined gene mutations.

**Conclusion:**

Azacytidine and B-cell lymphoma/leukemia-2 inhibitors have good efficacy and high safety in the treatment of AML and MDS, and the combined treatment is better than that of monotherapy, but the side effects of combination therapy are large.

## 1. Introduction

Acute myelogenous leukemia (AML) is a heterogeneous hematological malignancy characterized by clonal expansion of myeloid blast cells in peripheral blood, bone marrow, and/or other tissues [1, 2]. Clinical manifestations are mainly associated with inhibition of normal hematopoietic function and abnormal primitive and naïve cell infiltration of extramedullary tissues and organs, and the typical symptoms are fever, bleeding, anemia, hepatosplenomegaly, and lymphadenopathy. Myelodysplastic syndromes (MDS) are bone marrow stem cell diseases characterized by ineffective hematopoietic function, pancytopenia, and progressive bone marrow failure that have been discovered with the development of AML. According to statistics, the median age of patients diagnosed with AML is 68 years, while the median age of patients with confirmed MDS is more than 70 years [3].

Therefore, with the aging of the population, the incidence of the two is gradually increasing. Azacytidine and B-cell lymphoma/leukemia-2 inhibitors are demethylated drugs belonging to cytosine nucleotide analogues that kill tumor cells by inducing DNA demethylation and direct cytotoxic effects on bone marrow hematopoietic cells. Azacytidine is recommended for first-line treatment in elderly AML patients who are not suitable for intensive treatment regimens, and some studies have shown a combination of azacytidine and B-cell lymphoma/leukemia-2 inhibitors. Compared with other approved therapies, azacytidine and B-cell lymphoma/leukemia-2 inhibitors can prolong the overall survival to a similar or greater extent and are less toxic [4]. There are reports of clinical experience and results of the use of azacytidine and B-cell lymphoma/leukemia-2 inhibitors similar to those seen in clinical trials. All in all, azacytidine and B-cell lymphoma/leukemia-2 inhibitors abroad have been used as first-line drugs for the treatment of AML and high-risk MDS, while the domestic is currently mainly used to treat high-risk intermediate-risk-2 MDS in the international prognostic scoring system of patients with AML and chronic myelogenous leukemia.

In recent years, some new drugs targeted therapy for AML have been listed [5, 6] as FMS-like tyrosine kinase 3 inhibitors, sorafenib, and platelet-derived growth factor receptor a/0 (PDGFRa/0) inhibitor. Crenolanib has yielded good results in clinical trials of AML. In a variety of AML-targeted therapies [7], direct stimulation of the mitochondrial apoptosis pathway of cancer cells is a new therapeutic strategy. This pathway is regulated by the Bcl-2 gene protein family, which overexpresses tumor cells to evade apoptosis and become resistant to a variety of antineoplastic drugs [8]. Inhibiting the expression of Bcl-2 family proteins inhibits the formation of tumor neovascularization, thereby inhibiting tumor metastasis. Therefore, targeting Bcl-2 family proteins can inhibit tumor occurrence, development, and drug resistance, and Bcl-2 inhibitors become novel drugs that induce apoptosis of tumor cells. This article has reviewed the research progress of Bcl-2 inhibitors in AML-targeted therapy.

## 2. Information and Methods

### 2.1. General Information

In 2018.10-2021.02, our hospital clearly diagnosed AML/MDS which applies azacytidine and B-cell lymphoma/leukemia-2 inhibitors. Of the 31 patients treated, the cell smear method was used to detect bone marrow cell morphology, flow cytology to detect immunophenotyping, cell culture to detect cytogenetics, and second-generation sequencing to detect molecules. PCR fusion genes are detected by the method: Patient-Based 2016 WHO-AML/WHO-MDS Diagnostic Criteria Guidelines [9]. The prognosis grouping is based on the revision of the International Prognosis Scoring System (IPSS-R).

The inclusion criteria were as follows: (1) patient age 218 years, (2) at least 2 courses of chemotherapy, and (3) confirmed diagnosis 2016 WHO Diagnostic criteria guidelines.

The median age of 31 patients was 63 (29-86) years, with AML 18 cases and MDS 13 cases: 13 males and 18 females, 21 cases over the age of 60 years (260), and 10 cases below 60 years of age (<60 years); 2016 WHO-AML/WHO-MDS Diagnostic Criteria for typing were as follows: M5b 11 cases, M2a 5 examples, M4a 1 case, mixed cell type 1 case, and MDS-EB-2 8 examples, MDS-EB-1 5 cases. MDS Reference IPSS-R Grouping were as follows: 1 case in the very low-risk group, 3 cases in the low-risk group, 4 cases in the medium-risk group, and 5 cases in the high-risk group. In addition, 15 cases were detected for genetic mutations by second-generation sequencing [10]. This study obtained the consent of the patient and his/her family and signed the Informed Information Form, which was also proved by the ethical committee of people's Hospital of Leshan.

### 2.2. Treatment

31 patients with azacytidine and B-cell lymphoma/leukemia-2 inhibitor monotherapy or combination chemotherapy include 22 cases of Vidasa (Baxter Oncology GmbH, registration number H20170238, specification 100 mg/bottle) and 9 cases of Weishou (produced by Chia Tai Tianqing Pharmaceutical Group Co., Ltd., registration certificate number H20193278, specification 100 mg/bottle), which has the total dose of 75 mg/m^2^^∗^7 d, divided into 7-10 days of continuous subcutaneous injection, every 28-30 days for 1 course. There were 20 cases of monotherapy and 11 cases of combination therapy, including 4 cases of combined thalidomide and ubenemex, 2 cases of ubenmez, half of HAG cytidine, high spinel, and recombinant human granulocyte colony stimulator, and lenalidomide, venetok, cytarabine, dasatinib, and vermatinib mesylate of 1 case each [11]. During the treatment process, effective measures such as symptomatic stomach preservation, heart preservation, liver protection, alkalinization, and prevention of vomiting are also given to support and prevent; when hemoglobin V60 g/L, the infusion of filtered white red blood cell suspension is given as appropriate, and when the platelet count is V20^∗^10^9^/L, platelet transfusion and hemostatic sensitivity are appropriate to prevent bleeding; when infectious symptoms such as fever occur, routine improvement is routinely perfect CRP, procalcitonin, and blood bacteria cultures of both upper extremities, along with symptomatic antipyretics and antibiotic anti-inflammatory therapy [12].

### 2.3. Indicators and Efficacy and Safety Assessment

Adopted in fiscal 2006 MDS International Clinical Working Group (IWG 2006), efficacy evaluation criteria are judged, which mainly include complete remission (complete remission, CR), partial mitigation (partial remission, PR), bone marrow remission (marrow CR, mCR), hematology improved (hematological improve, HI) disease stabilization, and treatment failure: (1) CR: blast cells in the bone marrow < 5.0% simultaneously satisfy all cell lines with normal, peripheral blood neutrophil counts 21.0^∗^10^9^/L, hemoglobin 2110 g/L, platelet count 2100^∗^10^9^/L, and blast cells 0%; (2) mCR: the content of blast cells in the bone marrow < 5.0% decreases by 50.0% compared to before treatment, but if the peripheral blood reaches HIS, it could also be indicated; (3) PR: absolute peripheral blood values should be maintained for at least 2 months, with other requirements meeting the criteria for complete remission (in patients who are abnormal before treatment), but the total number of blast cells in the bone marrow is only 50.0% less than the overall number before treatment and still exceeds 5.0% regardless of the degree and morphology of cell proliferation; and (4) CR or PR recurrence after recurrence: at least one of the following should be included: (1) the proportion of bone marrow blast cells has returned to the proportion before chemotherapy; (2) the decrease in hemoglobin exceeds 15 g/L or rely entirely on blood transfusions; (3) 250.0% reduction in platelet or granulocyte count compared to optimal efficacy; (5) disease stability does not meet the minimum criteria for partial remission, but there is no evidence of progression of the disease for at least 8 weeks; (6) treatment failure: the patient dies or progresses with disease while receiving treatment development includes exacerbation of decreased blood cells, an increase in the proportion of blast cells in the bone marrow or the development of more severe than before treatment FAB subtypes; (7) HI: patients are assessed for hematological improvement based on the results of blood cell analysis and a decrease in red blood cell transfusion; and (8) total remission rate (overall response rate, ORR) = (CR + PR + mCR)/total number of patients^∗^100%. Adverse reactions occur during chemotherapy, see WHO evaluation criteria for indexes for the evaluation of adverse drug reactions during acute and subacute chemotherapy [13], which mainly include hematological toxicity and nonhematogenous, blood toxicity mainly such as decreased white blood cells, platelets, granulocytes, and decreased hemoglobin; nonhematogenous has gastrointestinal tract, liver function damage, kidneys, bladder, heart and nervous system abnormal symptoms, and positive signs, for the results of genetic mutations, the basis IWG 2006 efficacy evaluation criteria, and comprehensive analysis of gene polymorphisms for azacytidine treatment AML/MDS effects of efficacy and prognosis.

### 2.4. Statistical Analysis

Continuous normally distributed data are expressed as the means ± SDs. Statistical calculations were carried out using SPSS statistical software. Multiple comparisons were analyzed via analysis of variance (ANOVA) with the Tukey-Kramer multiple comparisons test. *P* values <0.05 were considered significant.

## 3. Result

### 3.1. Information of the Patients of This Study

A total of 104 courses of treatment were completed in the 31 patients of this study, the median course was 3 (1–12), and 6 patients who did not complete 2 courses of treatment were not counted in the statistics. The remaining 25 patients completed a total of 98 courses, with a median treatment course of 3 (2–12), 9 patients completed 4 courses, and 2 patients completed 6 courses. After 2 sessions, the ORR was 72.0% (18/25), with 2 CRES (8.0%), 16 mCR (64.0%), 5 patients with HI, 5 disease stable (20.0%), and 2 treatment failures (8.0%). The ORR of MDS was 66.7% (8/12), with CR 1 case (8.3%), mCR 7 cases (58.3%), and partner. In 1 case of HI, 4 cases (33.3%) were stable, the ORR of AML was 76.9% (10/13), and the CR1 case (7.7%) was mCR. There were 9 cases (69.2%), 4 cases with HI, 1 case (7.7%) with stable disease, and 2 cases (15.4%) who failed treatment. ORR over 60 years of age was 66.7% (10/15), with 10 mCR patients (66.7%), 3 patients with HI, and 5 patients (33.3%) that were treated stably; younger than 60 years of age, treatment failed treatment with 80.0% (8/10) ORR, 2 cases (20.0%), 6 cases (60.0%), 2 cases with HI, and example (20.0%) (see Table 1). For young and middle-aged patients, 2 patients did not undergo hematopoietic stem cell transplantation due to death in the later treatment process, and the remaining 8 patients refused due to economic problems. After 4 courses of treatment, the ORR was 77.8% (7/9), with 7 cases of mCR, 3 cases with HI, 1 case of recurrence after HI, and 2 cases of stable disease. After 6 courses of treatment, there were 2 cases of mCR and 1 case with HI. Followed up to 1 February 2021, the death toll was 10, the mortality rate was 40.0% (10/25), the median survival time was >5 (3–22) months, MDS and AML median survival was 8 (3–22) and 11 (3–19) months, respectively, and median survival times were 7 (3–22) and 11.5 (3–17) months at over and below 60 years. During 25 patients who received 2 courses of chemotherapy, 16 patients required blood transfusion products for support treatment, and the transfusion dependence rate reached 64%; during 9 patients receiving 4 courses of chemotherapy [14], only 5 patients needed blood transfusion products, and the transfusion dependence rate reached 55.5%.

### 3.2. Prognosis of Azacytidine and B-Cell Lymphoma/Leukemia-2 Inhibitors in the Treatment of MDS/AML

Among the 25 patients counted in this study, 14 were treated with monotherapy, with ORR of 64.3% (9/14), CR was 2 (14.3%), mCR was 7 (50.0%), and HI was 2. In patients, 2 patients (14.3%) have stable disease (21.4%), median survival time was 7.25 (3–19) months, 11 patients have combined therapy, ORR was 81.8% (9/11), mCR9 (81.8%), with HI three patients, and 2 patients with stable disease (18.2%), and the median survival time was 9 (4.5-22) months. In 8 cases treated with AML monotherapy, the ORR was 62.5% (5/8), CR was 1 case, mCR was 4 cases, and the patient was accompanied by HI with 2 patients, 1 patient with stable disease, 2 patients with treatment failure, median survival time of 6.25 (3–17) months, and 5 patients with combined therapy, ORR was 100% (5/5), and mCR5 patients. In 2 cases of HI, the median survival time was 13 (8.5-19) months. MDS monotherapy was 6 patients, ORR was 66.7% (4/6), CR was 1 case, mCR was 3 cases, disease stabilization have 2 patients, and median survival is 7.75 (4.5-22) months; 6 patients were treated with a combination of 6 cases, ORR was 66.7% (4/6), mCR was 4 cases, and 1 case was accompanied by HI [15].

The disease was stable in 2 cases with a median survival time of 10 (3–19) months. Based on disease typing analysis, MDS-EB-1 was 4 cases, ORR was 75.0% (3/4), CR was 1 case, mCR was 2 cases, and accompaniment was HI1. In one case, the median survival time was 11.5 (6–22) months for 1 case with disease stabilization, the MDS-EB-2 was 8 cases, the ORR was 62.5% (5/8), and the mCR was 5. In 3 cases, the disease was stable, and the median survival time was 6.5 (3 to 19) months. AML-M2a was 3 patients, ORR was 66.7% (2/3), mCR was 2 patients, treatment failure was 1 patient, the median survival time was 3 (3–14) months AML-M5b was 8 cases, ORR was 75.0% (6/8), CR was 1 case, and mCR was 5 cases, with HI 3 cases, one patient was stable, one patient was treated failed, and the median survival time was 12 (3–17) months, see Table 2.

### 3.3. Gene Mutations of Azacytidine and B-Cell Lymphoma/Leukemia-2 Inhibitors in the Treatment of MDS/AML

Fifteen patients were tested for gene mutations by second-generation sequencing, and the results were 14 combined mutations, including 11 TET2 mutations, 6 ASXL1 mutations (5 combined TET2 mutations), NPM1, and DNMT3A. There were 4 cases of mutations, there were 3 cases of U2AF1, NRAS, and IDH2 mutations, there were 2 cases of RUNX1, IDH1, and IDH1 CEBPA, FLT3-ITD and GATA mutations each in 2 cases: ETV6 and SF3B1, and there was 1 mutation each of KRAS, SETBP1, BCOR, PHF6, and MLL. TET2 mutation ORR was 54.5% (6/11), CR was 2 patients, mCR was 4 patients, with HI. In 2 cases, 4 patients were stable, and 1 patient failed treatment; ASXL1 mutation ORR was 66.7% (4/6), CR was 1 patient, and mCR was 3 cases. In 1 case, with 1 case of HI, 1 case of disease stabilization, and 1 case of treatment failure, TET2 with ASXL1 mutation ORR was 80.0% (4/5). 1 case of CR, 3 cases of mCR, 1 case with HI, and 1 case of stable disease were as follows. As of February 1, 2021, the above median survival times were 13 (3–22), 11 (8.5-22), and 13 (8.5-22) months, respectively. There were 9 cases of MDS comutation, ORR was 55.5% (5/9), CR was 1 case, mCR was 4 cases, with HI 1 patient, disease stable 4 patients, median survival time > AML comorbid mutation 5 patients, ORR of 60.0% (3/5), mCR 3 patients with 1 case of HI, and 2 cases of treatment failure, and the median survival time was 13 (3–14) months, see Table 3.

## 4. Discussion

AML is predominantly occurring in older adults and is mostly unsuitable for intensive therapy, due to a variety of poor prognostic factors, including a high proportion of poor cytogenetics, changes associated with myelodysplastic abnormalities, a high ECOG-PS score, and a combination of severe underlying disease [16]. The active ingredient of azacytidine and B-cell lymphoma/leukemia-2 inhibitors binds to RNA and DNA by interfering with RNA transcription and DNA of actively proliferating cells. Methyltransferase I is active and exerts its cytotoxic effect. Initially, it was thought that the main antitumor activity of azacytidine and B-cell lymphoma/leukemia-2 inhibitors was to interfere with nucleic acid metabolism and has a direct cytotoxic effect. Subsequently, however, azacytidine and B-cell lymphoma/leukemia-2 inhibitors have been shown to have preferential toxicity to proliferating malignant tumor cells but no toxic effect on normal cells. Subsequent studies have found that azacytidine and B-cell lymphoma/leukemia-2 inhibitors have other anticancer effects in addition to direct cytotoxicity, the most notable of which include targeting DNA hypermethylation, which is thought to help inhibit tumorigenesis and disrupt the maturation and differentiation of bone marrow cells [17]. In the pharmacokinetic study of azacytidine and B-cell lymphoma/leukemia-2 inhibitors, since the drug is only effective in proliferating cells and does not accumulate, a shorter treatment time per week is unlikely to cause azacytidine and B-cell lymphoma/leukemia-2 inhibitors to encounter at S Phase of all malignant cloned cells, which will demonstrate a higher efficacy with longer treatment per cycle [18].

The ORR of the two courses of this study was 72.0%, the median survival time was 8.5 months, the ORR of MDS and AML was 66.7% and 76.9%, respectively, and the median survival time was 8 and 11 months, respectively, suggesting that azacytidine improved the overall response rate of patients. It prolongs a certain amount of survival time. In a Canadian CCO study on the efficacy of azacytidine on AML/MDS, the ORR was 28.0%, and the median survival time was 11.6 months [19]. AZA-001 studies showed that azacytidine and B-cell lymphoma/leukemia-2 inhibitors had an ORR of 29.0% and a median survival of 24.5 for treatment of high-risk MDS months; AZA-AML-001 study [16] shows ORR in the treatment of AML patients with azacytidine and B-cell lymphoma/leukemia-2 inhibitors. At 27.8%, the median survival time was 10.8 months, which was an improvement in response rate compared with traditional supportive care, and azacytidine significantly improved patients' objective response rate, survival rate, and clinical outcome. The primary survival time in this study is relatively short, which is inconsistent with the above foreign studies, mainly because some patients are enrolled late and the follow-up time is too short, and the follow-up time of 6 patients is only about 3 months. The total response rate of this study is higher than that of foreign studies, and the reasons for the analysis may be related to the following factors; first of all, the number of samples studied in this paper is too small; secondly, the selection of enrollment objects is different, the CCO study enrollment objects are IPSS score medium-risk-2 and high-risk MDS and bone marrow blastocyst ratio 20-30% of patients with AML, and the patients enrolled in this article only need to meet the WHO 2016 diagnostic criteria, including patients with bone marrow blast cells > 30% and IPSS-R scores for each risk stratification; then, the length of treatment cycles varies, and this article only covers 2 courses, and 4 efficacy was evaluated after each session, with a median of 3 sessions compared with 6 and 9 for the CCO study and AZA-001, respectively. Again, the median age in the CCO study may be 74 years (19-99 years), possibly due to the difference in median age. AZA-001 is 69 years (42-83 years old) compared to the median age of 63 years (29-86 years) in this study; there may also be differences in treatment regimens, with 11 cases of combination therapy in this article resulting in a high overall response rate, compared with CCO and AZA-001. All patients enrolled in the group were monotherapy, but it did not exclude the difference in sensitivity to drugs and the difference in drug metabolism in domestic and foreign patients. The Rowe study [17] showed an ORR of 48.0% and a median survival time of 9.6 months, concluding that azacytidine appeared to be right WHO-AML has a good efficacy; although, IWG 2006 is not currently considered the standard form of AML efficacy assessment, but disease stabilization and HI are considered to continue to be used criteria for efficacy of azacytidine and B-cell lymphoma/leukemia-2 inhibitor therapy. In this paper, the ORR was 72.0% after 2 courses and 77.8% after 4 courses, indicating that the effective rate of patients increased with the prolongation of the treatment cycle, which is consistent with foreign related studies [18]. Azacytidine and B-cell lymphoma/leukemia-2 inhibitors' long-term chemotherapy can significantly improve patient survival outcomes. And patients with CR and PR should be appropriately extended chemotherapy, and treatment should be continued as long as the patient continues to benefit. In this article, the ORR for MDS is 66.7%, the ORR for AML is 76.9%, and the results show AML. The overall response rate was higher than that of MDS, indicating that the efficacy of azacytidine in the treatment of AML may be better than that of MDS, but the results of this study are inconsistent with the above domestic and foreign studies. The main reason may be that the sample size in this article is too small to cause the results to be different. Finally, the ORR of MDS-EB-1 in this paper was 75.0%, with a median survival time of 11.5 months and ORR of MDS-EB-2. It was 62.5% with a median survival time of 6.5 (3–19) months, suggesting that azacytidine and B-cell lymphoma/leukemia-2 inhibitors may be more effective than MDS-EB-2 in the treatment of MDS-EB-2. This seems to be consistent with the results of the study of Pichler et al. abroad. Therefore, azacytidine and B-cell lymphoma/leukemia-2 inhibitors are more effective in the treatment of AML/MDS [20].

In this study, the ORR of azacytidine and B-cell lymphoma/leukemia-2 inhibitor was 64.3%, the median survival time was 7.25 months, the ORR of the combination was 81.8%, and the median survival time was 9 months. Among them, AML single-agent ORR was 62.5%, median survival time was 6.25 months, combined ORR was 100%, and median survival time was 13 months. The ORR was 66.7%, the median survival was 7.75 months, the combined ORR was 66.7%, and the median survival time was 10 months. For adverse reactions, the incidence of hematoxicity of grades III-IV was 90.9% during combination therapy, and there were 3 cases of lung infection, 5 cases of liver function impairment, 2 cases of renal function impairment, 7 cases of hypoalbuminemia, and 2 cases of hyperuricemia; during monotherapy, the incidence of grade III-IV hematoxicity was 85.7%, and there were 3 cases of lung infection, 2 cases of liver function impairment, 1 case of renal function damage, and 3 examples of hypoalbuminemia. As can be seen above, the combined treatment of azacytidine and B-cell lymphoma/leukemia-2 inhibitors may be more effective than monotherapy, but the side effects of combination therapy are large, and others have found the receiving azacytidine and B-cell lymphoma. Patients treated with leukemia-2 inhibitors in combination with venetoclax had a longer overall survival and a higher incidence of remission than patients treated with azacytidine and B-cell lymphoma/leukemia-2 inhibitors alone. The incidence of febrile neutropenia was higher in the group than in the control group [21]. There is one azacytidine and B-cell lymphoma/leukemia-2 inhibitor combined with thalidomide for the treatment of clinically advanced MDS, CMML, and AML. The results of the phase II study [21–23] ORR was 63.0%, the overall survival was 28.1 months, and the nonhematotoxicity was grade III or higher 85.0%, indicating that combination therapy is good and that treatment is tolerated. This paper is consistent with the conclusions of relevant foreign studies, and all reflect the combination of azacytidine and B-cell lymphoma/leukemia-2 inhibitors with good efficacy, but the drug toxicity is greater.

The TET2 gene is located on chromosome 4q24, and the ASXL1 gene is located in chromosome 20qll, both of which are involved in the epigenetic and regulation of DNA. ASXL1 encodes an internal nuclear protein of 1541 amino acids and has transcriptional functions, which typically causes the C-terminus of the protein upstream of pPhD to be truncated, resulting in loss of gene function. TET2, on the other hand, is involved in the epigenetic regulation of DNA through the conversion of 5-methylcytosine to 5-hydroxycytosine. Multiple studies have shown that mutations in genes such as TET2 and ASXL1 are factors of poor prognosis, significantly shortening progression-free survival (PFS) and overall survival. In an evaluation study on TET2 gene mutation prediction of responses of MDS patients to demethylated drugs, the results showed Bejar et al. and Itzykson. The findings of the two authors were consistent, with ORRs of 55.0% and 52.0%, respectively, and it was concluded that TET2 deletion appeared to make tumor cells more sensitive in vivo to azacytidine and B-cell lymphoma/leukemia-2 inhibitors. TET2 mutations are more likely to identify patients who respond to the demethylated drug cocozacyanin. In this study, the TET2 mutation ORR was 54.5%, the median survival time was 13 months, the ASXL1 mutation ORR was 66.7%, the median survival time was 11 months, and the results were more consistent with foreign countries, indicating that although prognosis is poor in patients with AML/MDS mutations in TET2 and ASXL1 genes, treatment with azacytidine and B-cell lymphoma/leukemia-2 inhibitors may improve overall response rates and median survival, patient outcomes, and quality of life. Thus, azacytidine and B-cell lymphoma/leukemia-2 inhibitors may improve efficacy in patients with AML/MDS with genetic mutations [22].

In this study, 25 patients had different degrees of bone marrow suppression during chemotherapy, the incidence of grade III-IV hematogenous toxicity was 88.0%, the incidence of grade II hematogenousness was 12.0%, and most of them significantly improved after symptomatic support therapy. All patients experienced nausea and vomiting, with 1 case developed constipation and 2 cases developed diarrhea, supplemented by symptomatic antiemetic, laxative, and antidiarrheal treatment, symptoms were relieved, and no further gastrointestinal symptoms were developed. Foreign studies by Pleyer et al. showed that the incidence of grade III-IV hematoxicity was 48.0%, and III-IV grade neutrophilia, thrombocytopenia, and hemoglobin decreases were 35.0%, 30.0%, and 28.0%, respectively; the most common nonhemotoxicity was fatigue, gastrointestinal manifestations, unexplained pain, and erythema at the injection site. In this paper, 13 patients had fever, including 6 cases of fever with lung infection, the infection rate was 24.0%, the symptoms were basically alleviated after antibiotic treatment, and the chest CT showed that the inflammation was significantly reduced compared with before. The infection rate of the foreign AGMT research group was 33.0%, which was mainly manifested by pulmonary infection, sepsis, and other fever with unclear etiology, which was significantly higher than the results of this study. A systematic review and meta-analysis showed that the use of azacytidine and B-cell lymphoma/leukemia-2 inhibitors was associated with an increased risk of decreased neutrophil counts and platelet counts in patients with MDS/AML, and that azacytidine and B-cell lymphoma/leukemia-2 inhibitors did not significantly increase high anemia, leukopenia, or febrile neutrality compared with traditional supportive care risk of agranulocytosis [22]. In this study, 3 cases of renal function impairment and 7 cases of liver function damage appeared, and foreign studies found that adverse reactions such as elevated serum creatinine occurred during the application of azacytidine and B-cell lymphoma/leukemia-2 inhibitors; so, biochemical indicators such as liver and kidney function should be closely monitored during the chemotherapy process [23]. Nonhematogenousness is found to cause patients to develop symptoms of the heart system, mainly manifested as left ventricular failure, arrhythmias, hypertension, myocardial infarction, and angina. However, the above adverse reactions in the heart did not occur in this paper; therefore, in the treatment process, it is also necessary to improve the ECG and cardiac color ultrasound and monitor the cardiac enzyme profile and brain natriuretic peptides and other cardiac indicators. The transfusion dependence rate in 2 sessions of this study was 64.0%, and the transfusion dependence rate in 4 sessions was 55.5%. The results of the CCO study showed that the transfusion dependence rate of 354 patients receiving less than 4 cycles of treatment was 73.2%, the transfusion dependence rate of 692 patients receiving more than 4 cycles of treatment was 60.0%, and it was concluded that with the prolonged chemotherapy cycle time, the transfusion dependence rate of patients decreased and the safety increased. Therefore, azacytidine and B-cell lymphoma/leukemia-2 inhibitors are better off in the treatment of AML/MDS [24, 25].

## 5. Conclusion

In summary, the treatment of azacytidine and B-cell lymphoma/leukemia-2 inhibitors in AML/MDS can improve certain efficacy and has good safety, and the combination treatment is better than that of single drugs, but the side effects of combination drugs are large. However, the number of cases studied in this paper is small, and the sample size needs to be increased to further investigate the efficacy and safety of azacytidine and B-cell lymphoma/leukemia-2 inhibitors.

## Figures and Tables

**Table 1:** Information of patients of this study.

Courses of treatment	Patients	Median course	HI	Disease stable	Treatment failures
104	31	3 (1-12)	5	5	2

**Table 2:** Baseline features of 25 patients with AML/MDS.

Serial number	Gender	Age	FAB classification	IPSS-R	Score ECOG score	Transfusion dependence	Previous treatment
1	Man	71	M4a	—	1	Not	Not
2	Man	75	M5b	—	4	Not	Not
3	Woman	59	Hybrid	—	3	Be	Not
4	Woman	55	M5b	—	1	Be	Not
5	Woman	29	M2a	—	0	Be	Not
6	Woman	50	M5b	—	2	Be	Not
7	Woman	68	M5b	—	2	Be	Not
8	Woman	68	M5b	—	1	Not	Not
9	Man	45	M5b	—	1	Not	Not
10	Woman	62	M5b	—	1	Be	Not
11	Woman	58	M5b	—	0	Not	Not
12	Woman	63	M2a	—	1	Be	Not
13	Woman	80	M2a	—	2	Not	Not
14	Woman	64	MDS-EB-2	Risk	4	Be	Not
15	Woman	66	MDS-EB-2	Very low risk	2	Be	Not
16	Man	67	MDS-EB-1	Low risk	1	Not	Not
17	Man	68	MDS-EB-2	Medium-risk	1	Be	Not
18	Man	73	MDS-EB-2	Low risk	1	Be	Not
19	Man	53	MDS-EB-1	Medium-risk	2	Not	Not
20	Woman	57	MDS-EB-2	Risk	4	Be	Not
21	Woman	71	MDS-EB-1	Risk	3	Be	Not
22	Woman	60	MDS-EB-2	Medium-risk	3	Not	Not
23	Man	51	MDS-EB-1	Risk	2	Be	Not
24	Woman	65	MDS-EB-2	Low risk	1	Be	Not
25	Man	48	MDS-EB-2	Risk	3	Be	Not

**Table 3:** Comparison of reported results of azacytidine and B-cell lymphoma/leukemia-2 inhibitors in the treatment of MDS/AML.

Test code name	Number	Of patients of median age pa		Total response rate/%	Median survival time/month
		/years	/people		
This article investigates	AML/MDS	63	31	72.0	8.5
AZA-001	High-risk MDS	70	179	29.0	24.5
AZA-AML-001	265 years old AML	75	241	27.8	10.8
CCO	High-risk MDS/AML	74	1101	28.0	11.6
Pleyer	High-risk MDS/AML	73	302	48.0	9.6

## Data Availability

The data used to support this study is available from the corresponding author upon request.
